# Vacuolar sequestration capacity and long-distance metal transport in plants

**DOI:** 10.3389/fpls.2014.00019

**Published:** 2014-02-04

**Authors:** Jia-Shi Peng, Ji-Ming Gong

**Affiliations:** ^1^National Key Laboratory of Plant Molecular Genetics, Institute of Plant Physiology and Ecology, Shanghai Institutes for Biological Sciences, Chinese Academy of SciencesShanghai, China; ^2^National Center for Gene Research, Institute of Plant Physiology and Ecology, Shanghai Institutes for Biological Sciences, Chinese Academy of SciencesShanghai, China

**Keywords:** vacuolar sequestration capacity, vacuole, transporter, chelator, metal transport

## Abstract

The vacuole is a pivotal organelle functioning in storage of metabolites, mineral nutrients, and toxicants in higher plants. Accumulating evidence indicates that in addition to its storage role, the vacuole contributes essentially to long-distance transport of metals, through the modulation of Vacuolar sequestration capacity (VSC) which is shown to be primarily controlled by cytosolic metal chelators and tonoplast-localized transporters, or the interaction between them. Plants adapt to their environments by dynamic regulation of VSC for specific metals and hence targeting metals to specific tissues. Study of VSC provides not only a new angle to understand the long-distance root-to-shoot transport of minerals in plants, but also an efficient way to biofortify essential mineral nutrients or to phytoremediate non-essential metal pollution. The current review will focus on the most recent proceedings on the interaction mechanisms between VSC regulation and long-distance metal transport.

## INTRODUCTION

Mineral nutrients including iron (Fe), zinc (Zn), copper (Cu), manganese (Mn), nickel (Ni), and molybdenum (Mo) are required in different amounts by different plant tissues. Therefore, once taken up into plants, long-distance transport and allocation of these metals play a pivotal role in plant development and adaptation to the environment. To date, studies of long-distance root-to-shoot metal transport within plants focus preferentially on transporters localized to either xylem parenchyma cells or phloem companion cells, as they directly mediate xylem and phloem loading or unloading thus contributing essentially to this metal reallocation process. Moreover, some chelators, including nicotianamine (NA; reviewed by Curie et al., 2009), glutathione (GSH), and phytochelatins (PCs; reviewed by Mendoza-Cozatl et al., 2011), were observed to also act as important players in the process of long-distance transport of metals.

Plant vacuoles are predominant organelles serving as temporary storages for essential and toxic metabolites, mineral nutrients and toxic pollutants. Accumulating evidences indicate that in addition to the direct regulation from those ion transporters and chelators, the Vacuole sequestration capacity (VSC) also contributes substantially to long-distance transport and allocation of metals in plants. Vacuoles function as buffering pools where the sequestration capacities are dynamically adjusted to the changing environmental cues, through the interaction between tonoplast-localized transporters and ion chelators. This mini-review will focus on the regulation of VSC and its interaction with long-distance root-to-shoot transport of either essential or non-essential metals in plants.

## REGULATION OF VSC

### REGULATION BY TRANSPORTERS

Up to date, most tonoplast-localized metal transporters in plants (reviewed by Martinoia et al., 2012) have been identified to regulate VSC and hence metal allocation between different organs or tissues (**Table 1**).

**Table 1:** Tonoplast-located transporters that have impact on long-distance transport of metal micronutrients (or toxic metals) in plant.

Transporters	Mineral	Reference
MTP1	Zn	reviewed by Ricachenevsky etal. (2013)
MTP3	Zn	Arrivault etal. (2006)
ZIF1	Zn	Haydon and Cobbett (2007), Haydon etal. (2012)
NRAMP3/NRAMP4	Fe	Thomine etal. (2003), Lanquar etal. (2005)
VIT1/VIT2	Fe, Zn	Kim etal. (2006), Zhang etal. (2012)
FPN2(IREG2)	Fe, Co, Ni	Morrissey etal. (2009), Schaaf etal. (2006)
COPT5	Cu	Klaumann etal. (2011)
CAX2/CAX4	Cd	Korenkov etal. (2007)
HMA3	Cd	Ueno etal. (2010, 2011)

In response to mineral nutrient deficiency, genes involving in nutrient remobilization from vacuoles to cytosols, such as *NRAMP3* and* NRAMP4 *(Thomine et al., 2000, 2003), are up-regulated, thus reducing the VSC to release the stored nutrients and consequently alleviating nutrient deficiency. In contrast, other genes including *MTP3 *(*Metal Transporter 3*; Arrivault et al., 2006)*, ZIF1 *(*Zinc-Induced Facilitator 1*; Haydon and Cobbett, 2007)*, VIT2 *(*Vacuolar Iron Transporter 2*; Zhang et al., 2012)*, CAX4 *(*Cation Exchanger 4*; Mei et al., 2009), which regulate metal sequestration into vacuoles, are up-regulated when excessive metals are available in the environment, and the enhanced expression consequently leads to enlarge VSC and metal accumulation in vacuoles. Another group of genes including *VIT1*(Kim et al., 2006; Zhang et al., 2012)*, MTP1*(Kobae et al., 2004; Desbrosses-Fonrouge et al., 2005; Kawachi et al., 2009)*, COPT5* (*Copper Transporters 5*; Garcia-Molina et al., 2011; Klaumann et al., 2011), remain unaffected by the metal status in the environment, though functional abortion of these genes altered metal allocation at either subcellular or tissue levels, suggesting that a stable expression level of those genes enables proper metal allocation.

Metal hyperaccumulators modulate their VSC via a more conservative way than we have imagined, as they tend to utilize some transporters which are also present in their corresponding non-hyperaccumulators but have evolved with more complex regulation mechanisms. MTP1 is a key transporter modulating the VSC of Zn (Sinclair and Krämer, 2012; Ricachenevsky et al., 2013). Piled evidences suggest that the expression level of *MTP1* is greatly enhanced in various metal hyperaccumulators (Assunção et al., 2001; Persans et al., 2001; Becher et al., 2004; Dräger et al., 2004; Hammond et al., 2006; Talke et al., 2006; van de Mortel et al., 2006; Gustin et al., 2009; Shahzad et al., 2010; Zhang et al., 2011), which later on was shown to be attributable to genome amplification of gene copies, in contrast to a single copy in their relative non-hyperaccumulators (Dräger et al., 2004; Shahzad et al., 2010). A similar regulation of *TcHMA3* *(Heavy Metal ATPases 3)* was also observed (Ueno et al., 2011), among which gene amplification leads to much higher expression of *TcHMA3* in the accumulating ecotype Ganges of *Thlaspi caerulescens* than in the non-accumulating Prayon, thus VSC of Cd in roots is greatly reduced and more metal is driven to translocate to shoots.

### REGULATION BY CHELATORS

Phytochelatins are important chelating molecules in plants, which detoxify heavy metals via chelation and hence forming stable PCs-metal complexes which are subsequently sequestered into vacuoles (Cobbett and Goldsbrough, 2002). In an effort to identify the relative contribution to VSC by PCs and GSH, the authors unexpected found that when ectopically expressing *SpHMT1*, a fission yeast gene encoding vacuolar PC-Cd transporters, the rate of long-distance Cd transport was significantly delayed in *Arabidopsis* (Huang et al., 2012). They assumed that this delay might be due to the enlarged VSC in root vacuoles. To test their hypothesis, SpHMT1 was targeted to roots and as expected, accumulation of Cd, Cu, and As in seeds was reduced up to 70% of the controls. These results show that VSC of heavy metals is essentially regulated by PCs.

Nicotianamine is another kind of metal chelator which is ubiquitously present in higher plants. Recent studies suggest that NA modulates the VSC of Zn and Fe and hence their distribution. In the hyperaccumulator *Arabidopsis halleri*, large amounts of NA is present in the root tissues and was proposed to essentially contribute to long-distance transport of Zn to shoots, as in the *AhNAS2*-RNAi plants with substantially reduced NA contents, much less Zn was observed in the xylem sap and shoots (Deinlein et al., 2012). Another research showed that overexpression of *AtZIF1* in *Arabidopsis* enhanced NA sequestration into vacuoles (Haydon et al., 2012), which consequently led to Fe overaccumulation in shoot tissues. The authors implicated that enhanced vacuolar NA sequestration depleted cytosolic NA, thus affected the intercellular mobility of Fe as Fe-NA complex (Haydon et al., 2012).

The amino acid histidine (His) was also identified to be functional in Ni detoxification and translocation in some Ni hyperaccumulators (Krämer et al., 1996; Kerkeb and Krämer, 2003; Krämer, 2010). Using a tonoplast transport assay strategy, Richau et al. (2009) found that when Ni was supplied as a Ni-His complex, a much higher uptake rate was observed in tonoplast vesicles derived from the hyperaccumulator than those from the non-hyperaccumulator* T. arvense*. Given high concentration of His was mainly found in* T. caerulescens* roots, and the level is about 10 times of that in *T. arvense* roots, they postulated that accumulation of His in *T. caerulescens* roots reduces the VSC of Ni by cytosolic chelation, thus promoting Ni transport and hyperaccumulation in shoots.

In general, VSC regulation by chelators could be classified into two categories: (1) the chelated metals are prone to translocation into vacuoles, thus enlarging VSC of certain metals; or (2) chelation of metals leads to reduced vacuolar sequestration and hence decreasing the VSC of certain metals. Root-targeted expression of *TaPCS1 *in *cad1-3* significantly enhanced root-to-shoot long-distance transport of Cd (Gong et al., 2003), and disruption of NA biosynthesis retained Zn in roots (Deinlein et al., 2012). All these studies suggest that chelation of metals by PCs or NA tends to promote long-distance metal transport, though the chelation is supposed to enlarge VSC to some extent. One possible explanation might be that the VSC regulated by chelators is also dependent on relevant transporters, as overexpression of SpHMT1, the PC-Cd complex transporter, successfully trapped Cd in roots (Huang et al., 2012), indicating a complex interaction between chelators and their transporters in the regulation of VSC.

## VSC REGULATES LONG-DISTANCE METAL TRANSPORT IN PLANTS

### VSC AND TRANSPORT OF MINERAL NUTRIENTS

Consistent with its major function in photosynthesis, most cellular Fe is found in the chloroplast. However, a substantial amount of this mineral nutrient is also stored in leaf vacuoles. Zhang et al. (2012) isolated two tonoplast-localized metal transporters OsVIT1 and OsVIT2 from rice. Ectopic expression of *OsVIT1* and *OsVIT2* genes partially rescued the Fe and Zn sensitive phenotypes and increased vacuolar Fe and Zn accumulation in yeast, suggesting a primary role for *OsVIT1* and *OsVIT2* is sequestering Fe/Zn into vacuoles across the tonoplast. *OsVIT1* and *OsVIT2* are highly expressed in rice flag leaves. Functional disruption of these two genes led to decreased Fe/Zn accumulation in flag leaves while enhanced accumulation in rice grains and phloem exudates of flag leaves and uppermost nodes. Meanwhile, no obvious changes were observed in either uptake or root-to-shoot transport of Fe/Zn between the mutants and the wild-type. These observations suggest that *OsVIT1* and *OsVIT2* play an important role in Fe and Zn long-distance translocation between source (flag leaves) and sink organs (seeds), via the modulation of VSC for Fe and Zn in flag leaves. In *Arabidopsis*, functional disruption of the tonoplast-localized Fe transporters AtVIT1 (Kim et al., 2006), AtNRAMP3 (*Natural Resistance Macrophage Protein 3*) and AtNRAMP4 (Lanquar et al., 2005) resulted in growth arrest especially in Fe deficient condition, providing further support to the hypothesis that modulation of VSC essentially affect Fe mobilization and reallocation between different tissues in plants.

The hypothesis also applies to the modulation of the VSC of Zn in plants. *AtMTP3* mediates Zn transport into vacuoles and expresses preferentially in *Arabidopsis* roots. When exposed to excessive Zn, *AtMTP3* is induced thus enhancing the VSC and consequently Zn sequestration into vacuoles in roots. It is believed that this mechanism helps to protect the most important organelles including chloroplasts through reduced long-distance transport of Zn to aerial tissues (Sinclair and Krämer, 2012). One supportive evidence came from the observation that more Zn accumulated in shoot tissues of the *atmtp3* mutant (Arrivault et al., 2006). Consistent results were obtained in the research of other Zn transporters such as the tonoplast-localized AtZIF1. *AtZIF1* overexpression lines showed decreased Zn accumulation in shoots and increased root-to-shoot ratios of Zn concentrations compared to the wild-type control (Haydon and Cobbett, 2007; Haydon et al., 2012), as would be expected according to the theory that Zn translocation could be mediated by VSC.

Additional supportive evidences came from Cu reallocation. *AtCOPT5* is expressed in root vascular tissues at high levels, and functions as a vacuolar Cu exporter. In the T-DNA-insertion mutant *atcopt5*, remarkably increased copper concentrations were observed in the vacuoles compared with those in the wild-type. Correspondingly, more Cu accumulated in roots and less in siliques and seeds of the mutant plants (Garcia-Molina et al., 2011; Klaumann et al., 2011).

### VSC AND TRANSPORT OF TOXIC METALS

Non-essential toxic metal(loid)s including Cd and As may lead to adverse effects on plants, mainly through the derived oxidative injuries or competitive inhibition of essential mineral nutrient. To protect the aerial parts which are active in photosynthesis and other important biological processes, plants have evolved sophisticated machineries in regulating metal distribution between roots and shoots, among which VSC also plays a very important role.

One example is about the rice *OsHMA3*, which has been correlated to Cd accumulation in rice shoots. Specifically, Ueno et al. (2010) found that a functional disrupted *OsHMA3* allele resulted in Cd overaccumulation in rice shoots. Further research revealed that OsHMA3 is localized to the tonoplast in rice roots, and it functions primarily to mediate Cd transport into vacuoles. Overexpression of the functional *OsHMA3* allele significantly decreased Cd accumulation in rice grains, while no apparent effect was observed on the accumulation of other essential micronutrients. These results suggest that the VSC in rice roots mediated by OsHMA3 contributes essentially to the long-distance transport of Cd from roots to shoots.

Another example is about the metal hyperaccumulators. In contrast to non-hyperaccumulators, hyperaccumulators show extraordinarily high accumulation of toxic metals in aerial parts without any visual effects (reviewed by Krämer, 2010). Interestingly, studies have suggested that VSC regulation also gets involved in both the long-distance transport of toxic metals and the detoxification mechanisms that render plants high tolerance to metals.**It was shown that the VSC for Zn in hyperaccumulator* T. caerulescens* roots is significantly decreased, compared to the non-hyperaccumulating relative *T. arvense*, which consequently drives more Zn to translocate from roots to shoots as indicated by the enhanced xylem loading of Zn in *T. caerulescens *(Lasat et al., 1998)*.* In different ecotypes of the *T. caerulescens*, it was also found that the efficiency of Cd loading to the xylem is highly correlated to the VSC for Cd in root cells (Xing et al., 2008). A similar correlation between metal translocation efficiency to shoots and its VSC in roots is also found in *Sedum alfredii, *another Zn/Cd hyperaccumulator found specifically in Southern China (Yang et al., 2006). These observations suggest metal transport regulated by VSC modulation might be a common mechanism in hyperaccumulators. In addition to the regulation on long-distance metal transport, VSC also functions on metal detoxification in hyperaccumulators, supportive evidences came from the results that a predominant proportion of shoot Cd was localized to vacuoles (Küpper et al., 1999, 2001; Krämer et al., 2000; Ma et al., 2005).

## CONCLUDING REMARKS AND FUTURE DIRECTIONS

Vacuoles, occupying over 80% of the cellular volume in vegetative tissues, are the largest organelles undergoing relatively less metabolisms, which makes it perfect for vacuoles to store chemical compounds and metal ions. However, their role in regulating long-distance root-to-shoot transport of metals has been largely ignored, though such a deduction is becoming more and more apparent with accumulating evidences. Here we proposed that VSC plays a role of “buffering pool” to dynamically mediate long-distance metal transport in plants. Generally the VSC of certain metal varies between different plant tissues to ensure proper metal distribution, e.g., the VSC of toxic metals is larger in roots than in shoots, thus an essential proportion of the toxic metals will be trapped in roots as we normally observe. When exposed to high levels of toxic metals, specifically when the VSC of a certain metal is used up an “overflow” mechanism as proposed (Gong et al., 2003) takes over and the excessive metal is subjected to long-distance root-to-shoot transport. In metal hyperaccumulators, however, greatly reduced VSC in roots has evolved, which greatly promotes long-distance metal transport from roots to shoots. We also reviewed the regulation mechanisms of VSC by tonoplast-localized transporters and ion chelators. we believe that the study of VSC would contribute not only to a better understanding of metal homeostasis and distribution, but also to an efficient biofortification of essential mineral nutrients and phytoremediation of non-essential toxic metals.

As a primary producer, plants provide a lot of mineral nutrients that are essential for human health. However, some of these nutrients in the edible parts of stable crops are often deficient or poorly bioavailable thus resulting in an unbalanced diet. Therefore, nutrient biofortification is of urgent and necessary importance. In addition to the traditional approaches that tackle these concerns by increasing the efficiency of nutrient uptake and bioavailability (reviewed by Hirschi, 2009), modulation of VSC might be a more efficient way, in which nutrient taken into plants are forced to accumulate in targeted tissues, thus enhanced uptake might not be required and the risk of undesired accumulation of toxic metals is greatly reduced (Arrivault et al., 2006; Haydon et al., 2012; Zhang et al., 2012). Furthermore, targeted modulation of VSC could also help to reduce toxic metal accumulation in edible tissues, as demonstrated by the root-specific expression of *SpHMT1* or the natural variation in *OsHMA3* in rice (Ueno et al., 2010; Huang et al., 2012), where a strong correlation between the VSC in roots and metal accumulation in shoots was observed.

On the other side, phytoremediation has been proposed as an efficient way to tackle the widespread heavy metal pollution in many countries, however, the practical application of metal hyperaccumulators to field trial is not so optimistic, mainly because of the relative low biomass and growth rate of those specialized plants. In these specific circumstances, an optimal alternative could be the fine modulation of the VSC in both roots and shoots in some plants with large biomass and growth rate.

## Conflict of Interest Statement

The authors declare that the research was conducted in the absence of any commercial or financial relationships that could be construed as a potential conflict of interest.
